The article "Naringin Alleviates Diabetic Kidney Disease through Inhibiting Oxidative Stress and Inflammatory Reaction" was retracted in 2018. Reasons: false authorship; lack of ethics approval or compliance; ethical violations by an author.

# Naringin Alleviates Diabetic Kidney Disease through Inhibiting Oxidative Stress and Inflammatory Reaction

**DOI:** 10.1371/journal.pone.0143868

**Published:** 2015-11-30

**Authors:** Fenqin Chen, Ning Zhang, Xiaoyu Ma, Ting Huang, Ying Shao, Can Wu, Qiuyue Wang

**Affiliations:** 1 Department of Geratology for Cadres, The First Affiliated Hospital of China Medical University, Shenyang 110001, People’s Republic of China; 2 Department of Pathphysiology, College of Basic Medical Sciences, China Medical University, Shenyang 110013, People’s Republic of China; 3 Department of Endocrine and Metabolic Diseases, The First Affiliated Hospital of China Medical University, Shenyang 110001, People’s Republic of China; University of Louisville, UNITED STATES

## Abstract

Naringin, a flavanone glycoside extracted from Citrus grandis Osbeck, has a wide range of pharmacological effects. In the present study we aimed at demonstrating the protective effect of naringin against diabetic kidney disease (DKD) and elucidating its possible molecular mechanism underlying. The beneficial effect of naringin was assessed in rats with streptozotocin (STZ)-induced diabetes and high glucose-induced HBZY-1 cells. According to our results, first we found that naringin relieved kidney injury, improved renal function and inhibited collagen formation and renal interstitial fibrosis. Second, we confirmed that naringin restrained oxidative stress by activating Nrf2 antioxidant pathway. Moreover, the results suggested that naringin significantly resisted inflammatory reaction by inhibiting NF- κ B signaling pathway. Taken together, our results demonstrate that naringin effectively alleviates DKD, which provide theoretical basis for naringin clinically used to treatment of DKD.

## Introduction

Diabetes is a metabolic disorder syndrome characterized by a chronically raised blood glucose level, which is caused by various kinds of factors including hereditary factor, immune dysfunction, microbial infection, energetic factor and so on[1]. Diabetes as a systemic metabolic disease, has a number of chronic or acute complications, such as diabetic kidney disease (DKD), retinopathy, hypertension, diabetic food and diabetic ketoacidosis[2]. DKD is the most common and severe chronic complication of diabetes and is also the major microvascular complication, which is morphologically characterized by excessive accumulation of the extracellular matrix and could ultimately progress to tubulointerstitial fibrosis[3, 4]**错误!超链接引用无效。错误!超链接引用无效。**. There is no symptoms of the early diabetes, and with the course of illness the incidence rate of DKD is increased. DKD is one of the main causes of death in diabetic patients. However, at present there are few effective treatment options for DKD, so the development of new therapeutic approaches will be of great importance in alleviating DKD and reducing the mortality rate of diabetic patients.

The article "Naringin Alleviates Diabetic Kidney Disease through Inhibiting Oxidative Stress and Inflammatory Reaction" was retracted in 2018. Reasons: false authorship; lack of ethics approval or compliance; ethical violations by an author.

Naringin, a flavanone glycoside, has many kinds of pharmacological activities, such as anti-inflammatory, antibacterial, and antineoplastic et al. Recently, the effect of naringin on alleviating diabetes and diabetic complications has been receiving increasing attention[5, 6]**错误!超链接引用无效。错误!超链接引用无效。**. Study by Xulu et al showed that naringin could ameliorate atherogenic dyslipidemia but not hyperglycemia in rats with type 1 diabetes[7]. In high fat fed/streptozotocin-induced type 2 diabetic rats, naringin could directly lower glucose levels and attenuate hyperglycemia-mediated oxidative stress and proinflammatory cytokine production[8]. Moreover, many studies have shown that naringin alleviated high glucose-induced injuries in cardiac cells[9, 10]**错误!超链接引用无效。错误!超链接引用无效。**. Recently, Kandhare et al found that naringin relieved diabetic foot ulcer in rats by promoting angiogenesis and inhibiting endothelial apoptosis[11]. However, the effects of naringin on DKD and the underlying mechanisms have not been fully understood.

This is the first time we investigated the protective effects of naringin against DKD and elucidated relative molecular mechanisms in STZ-induced diabetic rat model in vivo and high glucose-induced HBZY-1 cells in vitro.

## Materials and Methods

### Ethics statement

All animal experiments were carried out strictly in accordance with international ethical guidelines and the National Institutes of Health Guide concerning the Care and Use of Laboratory Animals. The experiments were approved by the Institutional Animal Care and Use Committee of China Medical University.

### Drugs and Antibodies

Naringin with purity of ≥ 95% was purchased from Sigma Chemical Co. (St Louis, USA) and dissolved in sterile normal saline as a stock concentration of 20 mg/ml and stored at −20°C in the dark. The chemical structural of naringin is showed in Fig 1. STZ was purchased from Solarbio Science and technology Co., Ltd (Beijing, China). STZ was dissolved in 0.1 M citrate buffer with a concentration of 32.5 mg/ml. The antibodies used in our study were as follows: Collagen I (Boster, China), MMP2 (Boster, China), TIMP-1 (Boster, China), TGF-β1 (Santa Cruz, USA), I κ B α (Bioss, China), p-I κ B α (Bioss, China), NF-κ B (Boster, China), Nrf2 (Boster, China), HO-1 (Santa Cruz, USA), β-actin (Santa Cruz, USA), Histone H3 (Bioss, China).

**Fig 1:** The chemical structure of naringin. The molecular formula of naringin is C27H32O14 and the molecular weight is 580.53.

The article "Naringin Alleviates Diabetic Kidney Disease through Inhibiting Oxidative Stress and Inflammatory Reaction" was retracted in 2018. Reasons: false authorship; lack of ethics approval or compliance; ethical violations by an author.

### Animals and Experimental Protocol

Male Sprague-Dawley rats (200-250g) were obtained from Beijing Vital River Laboratory Animal Co., Ltd. (Beijing, China). The animals were maintained at 23°C under a 12 h light-dark cycle with free access to standard pellet chow (60% carbohydrate, 20% protein, 4.5% fat, 5% fiber, 1.15% calcium, 0.85% phosphorus, 0.75% potassium, 0.3% sodium, 0.15% magnesium, 345 ppm iron, 20 IU/g vitamin A, 4 IU/g vitamin D, 45 ppm vitamin E, 20 ppm vitamin K, 70 ppm vitamin B1, 30 ppm vitamin B5, 1900 ppm choline, 80 ppm niacin, etc.) and water and monitored daily. The rats were randomly divided into six groups: control, naringin (80 mg/kg), STZ, STZ + naringin (20 mg/kg), STZ + naringin(40 mg/kg), STZ + naringin(80 mg/kg). The rats in the STZ and STZ + naringin groups were intraperitoneally injected with STZ (65 mg/kg). The control and naringin groups were intraperitoneally injected with 0.1 M citrate buffer of same volume. After injection of STZ for 3 and 5 days, blood glucose levels were measured by tail vein puncture blood sampling. The rats except in control and naringin groups with blood glucose levels >16.7 mM on both days were chosen for the following experiments while ensuring there were 6–8 rats in each group. Subsequently, the naringin and STZ + naringin groups were intraperitoneally injected with naringin at respective dosage every day for 12 weeks. An equivalent volume of sterile normal saline was intraperitoneally injected into rats in the other groups for 12 weeks. After 12 weeks treatment with naringin all the animals were euthanized by injection of sodium pentobarbital(50 mg/kg) and peripheral blood, urine and kidney tissues were collected for further tests. The body weight and dietary intake were measured before and at the end of the experiment. All animals were sacrificed by cervical dislocation.

### Cell Culture and Treatment

The rat glomerular mesangial cell line HBZY-1 was obtained from the Cell Collection Center, Wuhan university. HBZY-1 cells were cultured in DMEM (Gibco, USA) supplemented with 10% fetal bovine serum (Hyclone, USA), 100 μg/ml streptomycin and 100 U/ml penicillin (Hyclone, USA), under a 5.0% CO_2_ atmosphere, at 37°C. To investigate the beneficial effect of naringin in vitro, HBZY-1 cells were administered 10 μM naringin for 2 h prior to challenge with 30 mM glucose for 48 h.

### Biochemical Determination

The measurement of blood urea nitrogen(BUN), and creatinine(Cr) in peripheral blood was performed using commercially-available kits(Jiancheng biotech, China). The urinary protein level was detected by Bradford Protein Assay Kit(Beyotime, China), according to the manufacture’s instructions.

The article "Naringin Alleviates Diabetic Kidney Disease through Inhibiting Oxidative Stress and Inflammatory Reaction" was retracted in 2018. Reasons: false authorship; lack of ethics approval or compliance; ethical violations by an author.

### Histological Analysis

Rat kidney samples were fixed in 10% buffered formalin, sectioned and embedded in paraffin. 5 μ m kidney sections were prepared for routine periodic acid–schiff (PAS) and Masson’s staining. Renal histopathologic change was assessed by stained with PAS. The Masson’s staining was performed to observe the collagen formation in kidney. Under a microscope(Olympus, Japan), each section was randomly selected and photographed for 5 fields.

### Immunohistochemical Staining

The immunohistochemistry staining for collagen I expression in renal tissues was performed on formalin-fixed, paraffin-embedded samples. 5 μm sections were chosen and deparaffinized, rehydevrepated with graded xylene-alcohol then incubated with peroxidase blocking reagent to inhibit nonspecific binding. Then the sections were incubated with collagen I antibody at 4°C overnight and subsequently incubated with horseradish peroxidase-conjugated goat anti-rabbit secondary antibody for 30 min at room temperature. Using diaminobenzidine peroxidase substrate the result was visualized and counterstained with Mayer’s hematoxylin (Sigma, St. Louis, MO). Under 400x magnification, the sections were observed and photographed using a microscope.

### Measurement of Oxidative Stress

To evaluate oxidative stress injury, the malondialdehyde(MDA) levels, superoxide dismutase(SOD) and glutathione peroxidase(GSH-Px) activities, and ROS production were detected using commercially-available kits(Jiancheng Biotech, China), according to manufacturer’s instructions.

### ELISA

The levels of TNF-α, MCP-1, ICAM-1 and VCAM-1 in kidney tissues and cell culture supernatants were detected by commercially-available ELISA kits(Boster, China), according to manufacturer’s instructions. TNF-α, MCP-1, ICAM-1 and VCAM-1 concentrations were calculated by generating a standard curve using standard proteins and analyzed respectively.

### EMSA

The DNA binding activity of NF-κ B and Nrf2 in nucleus was measured by EMSA assay. Briefly, the nuclear protein was extracted in renal tissues with a nuclear extraction kit (Beyotime, China). Then using BCA protein estimation kit (Beyotime, China) the protein concentration was determined. Biotin-labeled oligonucleotide probes were then incubated with equal amounts of nuclear proteins for 20 min at room temperature. Then the samples were separated on a nondenaturing polyacrylamide gel at 180 V for 80 min. After electrophoresis, proteins were transferred to nylon membrane by electroblotting. After incubation with horseradish peroxidase-conjugated streptavidin, the UV-cross linked and biotin-labelled DNA was detected by chemiluminescence.

The article "Naringin Alleviates Diabetic Kidney Disease through Inhibiting Oxidative Stress and Inflammatory Reaction" was retracted in 2018. Reasons: false authorship; lack of ethics approval or compliance; ethical violations by an author.

### Western blot Assay

The kidney tissues and HBZY-1 cells from different groups were lysed in RIPA and denatured. After the determination of protein concentration by BCA protein estimation kit(Beyotime, China), equal quantities proteins samples were separated by SDS-PAGE, transferred to polyvinylidene fluoride and blocked with 5% non-fat dry milk in PBS. The membranes were incubated with anti-Collagen I(1:400), anti-MMP2(1:400), anti-TIMP-1(1:400), anti-TGF-β1(1:500), anti- I κ B α(1:500), anti- p-I κ B α(1:500), anti- NF-κ B(1:400), anti- Nrf2(1:400), anti-HO-1(1:200), anti-β-actin(1:1000), anti-Histone H3(1:1000) primary antibodies respectively, at 4°C overnight. The membranes were then incubated with goat anti-rabbit secondary antibody conjugated with horseradish peroxidase (1:5000). Results were visualized with ECL detection reagent(Beyotime, China).

### MTT Assay

Cell proliferation was assessed by MTT assay. Briefly, the HBZY-1 cells were plated into 96-well plates (Corning, USA) and pretreated with various concentrations(1, 5, 10, 25, 50, 100 μM) of naringin for 2 h. Then cells were treated with 30 mM glucose for 24 h. The control group was added sterile normal saline in the same volume. After treatment, all the wells were incubated with 20 μl of 5 mg/ml MTT (Sigma-Aldrich, USA) for 4 h at 37°C. Subsequently, 100 μl of DMSO were used to dissolve the formed formazan crystals after removal of the supernatant. The result was recorded at 490 nm on a microplate reader (Bio-Tek, USA).

### HO-1 Activity Detection

According to manufacturer’s instructions, the activity of HO-1 was measured by detecting bilirubin production using a commercially-available kit(Jiancheng biotech, China).

### Immunofluoresence Staining

HBZY-1 cells were seeded on cover slips. Followed by fixation with 4% paraformaldehyde for 30 min and permeabilization in 0.1% TrionX-100 for 15 min at room temperature. Then the cells were blocked with 5% BSA for 30 min at room temperature, and incubated with primary antibody against NF-κ B overnight at 4°C. After incubation with secondary antibody for 60 min at room temperature, the cover slips were washed with PBS and stained with DAPI. Under 400× magnification, images were randomly taken in 5 different microscopic fields by fluorescence microscope (Olympus, Japan).

### Statistical Analysis

All data are given as means ± SD. The significance of differences among experiment groups were analyzed by one-way ANOVA followed by a Bonferroni's Multiple Comparison Test using GraphPad Prism 5 software. A p-value of less than 0.05 was considered significant.

## Results

### Effects of naringin on renal morphology and kidney injury biochemical indexes in STZ-induced diabetic rats

As shown in Fig 2A, the pathological changes in kidney tissues were observed by PAS staining. Compared with control group, the glomerular and tubular injury was prominent in STZ-induced diabetic rats. Treatment with naringin significantly alleviated renal injury in diabetic rats. The body weights and food intake of rats and kidney injury biochemical indexes were assessed and shown in Fig 2B–2G. The body weights of diabetic rats were obviously decreased, while treatment with naringin could increase diabetic rats body weight significantly (P<0.05). The mean food intake, ratio of kidney weight/body weight and levels of BUN, Cr and UP were significantly elevated (P<0.05) in diabetic group compared with those in the control group, whereas in naringin treatment groups these indexes were reduced significantly.

The article "Naringin Alleviates Diabetic Kidney Disease through Inhibiting Oxidative Stress and Inflammatory Reaction" was retracted in 2018. Reasons: false authorship; lack of ethics approval or compliance; ethical violations by an author.

**Fig 2:** Naringin mitigated changes of pathomorphology and kidney injury biochemical indexes. (A) The pathological changes of renal tissues were investigated by PAS staining(400×). The glomerular injury and tubular injury scores were shown. (B) Body weight and percentage change in weight of rats. (C) Food intake per rat per day. (D) The ratios of kidney weight/ body weight were calculated. The concentrations of BUN (E), Cr(F), and UP(G) were detected. Results represent three independent experiments. Data were expressed as means ± SD, n = 6.^a-d^ Means with different superscripts are significantly different (P< 0.05).

### Naringin inhibits the collagen production in STZ-induced diabetic rats

The collagen production and renal interstitial fibrosis was observed by Masson’s staining. As shown in Fig 3A, administration of naringin effectively alleviated (P<0.05) the collagen deposition and renal interstitial fibrosis in diabetic rats. In addition, the results of western blot and immunohistochemical staining assay suggested that the protein level of collagen type I was up-regulated in diabetic rats compared with control group. However, treatment with naringin could reduce the protein level of collagen type I (Fig 3B and 3C). Moreover, the collagen production and degradation related proteins were assessed by western blot. As shown in Fig 3C, the protein expressions of TIMP-1 and TGF-β1 were increased and that of MMP-2 was decreased in diabetic rats compared with control group, whereas treatment with naringin could inhibit the changes of these proteins.

**Fig 3:** Naringin inhibited collagen production and renal interstitial fibrosis. (A) The collagen deposition and renal interstitial fibrosis was observed by Masson’s staining(200×). The percentages of fibrosis area were shown. (B) The expression of collagen I in kidney tissues was determined by immunohistochemical staining(400×). (C) The expressions of collagen I, MMP-2, TIMP-1 and TGF-β1 in kidney tissues were detected by western blot. Results represent three independent experiments. Data were expressed as means ± SD, n = 6.^a-c^ Means with different superscripts are significantly different (P< 0.05).

The article "Naringin Alleviates Diabetic Kidney Disease through Inhibiting Oxidative Stress and Inflammatory Reaction" was retracted in 2018. Reasons: false authorship; lack of ethics approval or compliance; ethical violations by an author.

### Naringin inhibits high glucose-induced rat mesangial cells proliferation

The proliferation of HBZY-1 cells was obviously promoted (P<0.05) by treatment with high glucose for 24 h compared with control group, which could be inhibited by pretreatment with naringin remarkably (Fig 4).

**Fig 4:** Naringin inhibited high glucose-induced proliferation in HBZY-1 cells. The proliferation of HBZY-1 cells was determined by MTT assay. Data were expressed as means ± SD, n = 5.^a-f^ Means with different superscripts are significantly different (P< 0.05).

### Naringin reduces oxidative stress induced by STZ *in vivo* and high glucose *in vitro*

To evaluate the oxidative stress injury, the levels or activities of MDA, SOD, GSH-Px, and ROS were determined. As shown in Fig 5A–5D, the levels of ROS and MDA were significantly elevated and activities of SOD and GSH-Px were reduced (P<0.05) in kidney tissues of diabetic rats or high glucose-induced HBZY-1 cells. However, treatment with naringin could result in decreased levels of ROS and MDA and increased activities of SOD and GSH-Px. Moreover, the expression and activity of Nrf2, the key regulator of the antioxidative signaling pathway, and its downstream target HO-1 was observed. As assayed by western blot and shown in Fig 5E, Nrf2 expression in the nuclei was increased induced by STZ in vivo and high glucose in vitro, which could be promoted by treatment with naringin. Moreover, the expression and activity of HO-1 was accordingly increased (P<0.05) by treatment with naringin (Fig 5E and 5G). As shown in Fig 5F, the DNA binding activity of Nrf2 was significantly increased by naringin treatment (P<0.05).

**Fig 5:** Naringin restrained oxidative stress injury by activating Nrf2 antioxidant pathway. The concentration of MDA (A), the activity of SOD(B) and GSH-Px(C) in kidney tissues were detected. Data were expressed as means ± SD, n = 6. (D) The ROS production in HBZY-1 cells was evaluated by flow cytometry and ROS generation rates were shown. Data were expressed as means ± SD, n = 3. (E) The protein levels of Nrf2 and HO-1 in kidney tissues or HBZY-1 cells were detected by western blot. Results represent three independent experiments. (F) The DNA binding activities of Nrf2 in kidney tissues were assessed by EMSA assay. Data were expressed as means ± SD, n = 5. (G) The HO-1 activities in kidney tissues were determined. Data were expressed as means ± SD, n = 6.^a-d^ Means with different superscripts are significantly different (P< 0.05).

The article "Naringin Alleviates Diabetic Kidney Disease through Inhibiting Oxidative Stress and Inflammatory Reaction" was retracted in 2018. Reasons: false authorship; lack of ethics approval or compliance; ethical violations by an author.

### Naringin inhibits inflammatory reaction induced by STZ *in vivo* and high glucose *in vitro*

To assess the effect of naringin on inflammatory reaction, some representative inflammatory markers and related molecules were measured by ELISA. As shown in Fig 6, the levels of TNF-α, MCP-1, ICAM-1 and VCAM-1 were obviously increased (P<0.05) both in diabetic rats and in high glucose treated HBZY-1 cells. However, the levels of these markers were decreased significantly by naringin treatment.

**Fig 6:** Naringin inhibited inflammatory reaction in kidney tissues and HBZY-1 cells. The TNF-α(A), MCP-1(B), ICAM-1(C) and VCAM-1(D) levels in kidney tissues were determined by ELISA assay. Data were expressed as means ± SD, n = 6. The TNF-α(E), MCP-1(F), ICAM-1(G) and VCAM-1(H) levels in HBZY-1 cells were determined by ELISA assay. Data were expressed as means ± SD, n = 3.^a-d^ Means with different superscripts are significantly different (P< 0.05).

### Naringin inhibits NF-κ B activation induced by STZ *in vivo* and high glucose *in vitro*

Western blot assay revealed that the expression of NF-κ B in the cytoplasm was decreased and that in the nuclei was increased in diabetic rats or high glucose treated HBZY-1 cells, which could be significantly reversed by naringin treatment (Fig 7A). The level of I κ B α protein was decreased and that of p-I κ B α was increased significantly induced by STZ or high glucose compared with control group. This change was significantly inhibited by naringin treatment. Subsequently, the distribution of NF-κ B was determined by immunofluorescence staining. As shown in Fig 7B, obvious distribution change of NF-κ B from cytoplasm to nucleus was induced by high glucose, whereas treatment with naringin significantly inhibited the distribution change of NF-κ B. To further confirm the effect of naringin on NF-κ B activation, the DNA binding activity of NF-κ B was detected by EMSA assay. As shown in Fig 7C, the DNA-binding activity of NF-κ B was increased (P<0.05) in diabetic rats compared with control group, which could be inhibited by treatment with naringin.

**Fig 7:** Naringin suppressed NF-κ B signaling pathway activation. (A) The protein levels of p-I κ B α, I κ B α and NF-κ B in kidney tissues and HBZY-1 cells were determined by western blot. Results represent three independent experiments. (B) The distribution change of NF-κ B in HBZY-1 cells was observed by immunofluorescence assay. Results represent three independent experiments. (C) The DNA binding activities of NF-κ B in kidney tissues were assessed by EMSA assay. Data were expressed as means ± SD, n = 5.^a-c^ Means with different superscripts are significantly different (P< 0.05).

The article "Naringin Alleviates Diabetic Kidney Disease through Inhibiting Oxidative Stress and Inflammatory Reaction" was retracted in 2018. Reasons: false authorship; lack of ethics approval or compliance; ethical violations by an author.

### Naringenin inhibites high glucose-induced proliferation, inflammatory reaction and oxidative stress injury in HBZY-1 cells

To further confirm the effect of naringin, additional experiments on naringenin, the aglycone and also one of important in vivo metabolites of naringin, was performed. As shown in S1B Fig, 5 μM naringenin could significantly restrain high glucose-induced proliferation of HBZY-1 cells. The effective concentration of naringenin was lower than that of naringin. Moreover, the representative inflammatory markers and molecules were measured by ELISA. As shown in S1C–S1F Fig, the levels of TNF-α, MCP-1, ICAM-1 and VCAM-1 induced by high glucose were decreased significantly by naringenin treatment. The level of ROS induced by high glucose was decreased by naringinin (S1G Fig). In addition, western blot assay revealed that the increased expression of NF-κ B in the nuclei and decreased expression of NF-κ B in the cytoplasm induced by high glucose was reversed by naringenin treatment. The expression of HO-1, Nrf2 in nuclei and cytoplasm was changed by treatment with naringenin in the same manner as naringin (S1H Fig).

## Discussion

Given DKD does great harm to human, selecting and identifying effective drugs on prevention and treatment of DKD has been the hot research. In this study, we focused on investigating the protective effects of naringin, a bioactive glucoside of pomelo (Citrus grandis Osbeck) widely applied to food, pharmaceutical and cosmetic, and elucidated the potential molecular mechanisms. The highest dose of naringin in this study is roughly equivalent to 100 g citrus fruits, which is close to normal daily human intake. Mullen et al. reported that the glucosides can be existed by glucosyltransferase in kidney [12]. So the research of naringin against kidney injury induced by diabetics has strong realistic meaning. Our study finds some new interesting information about naringin treatment alleviating DKD via in vivo and in vitro studies. This is the first time that naringin has been reported to have protective effect on DKD.

DKD is one of the most common microvascular complications and is also the main cause of chronic renal failure. The main pathological feature of DKD is extracellular matrix (ECM) accumulation, which could result in glomerular sclerosis accompanied by proteinuria, edema and hypertension. The basement membrane and ECM are mainly consist with collagen, fibronectin and laminin[13]. MMP-2 is one of important ECM-degrading enzymes. Under physiological condition, MMP-2 and TIMP-1 participate in maintaining the balance of ECM production and degradation. In the course of DKD, the transcription of TGF-β1 is promoted and the synthesis of collagen I protein is increased, which causes basement-membrane thickening, glomerulus hypertrophy and glomerulosclerosis. In our present study, DKD model was produced by intraperitoneal injection with STZ in rats and the results showed that naringin could effectively improve renal function, decrease collagen formation and ECM accumulation by regulating MMP-2, TIMP-1 and TGF-β1 expression.

The article "Naringin Alleviates Diabetic Kidney Disease through Inhibiting Oxidative Stress and Inflammatory Reaction" was retracted in 2018. Reasons: false authorship; lack of ethics approval or compliance; ethical violations by an author.

The pathogenesis of DKD is complicated involving various factors and signal pathways. However, increasing evidence has confirmed that oxidative stress played key roles in the development of DKD[14, 15]**错误!超链接引用无效。错误!超链接引用无效。**. Kidney is one of the most sensitive organs to oxidative stress and could be injured by reactive oxygen species (ROS) directly. In hyperglycemic state, ROS production is induced by various factors, which activates many signal transduction pathways by interacting with lipids, proteins, and DNA[16]. In addition, high glucose also affects the ability of kidney cells to clear the oxygen free radical[17]. For example, the activities of SOD, GSH-Px and other anti oxidases are decreased in DKD. Given the importance of oxidative stress in the progression of DKD, the antioxidant therapy of DKD has increasingly become the hot spot in basic researches and clinical studies. A previous study found that vitamin E and vitamin C could inhibit the oxidative stress and renal glomerular basement membrane thickening in diabetic kidney[18]. Bhatti et al found that alpha-lipoic acid could alleviate glomerular sclerosis and interstitial fibrosis by inhibiting oxidative stress in STZ-induced DM rats[19]. Our results were consistent with previous studies and demonstrated that naringin remarkably alleviated oxidative stress injury in vivo and in vitro.

A complex antioxidant defense system is formed in the body to fight free-radical damage. The expressions of protective proteins are induced to relieve the tissue damage in oxidative stress status. Nrf2 could play an important role in anti-oxidative stress and the activation of it is tightly regulated by intracellular signaling pathways. Under the physiology condition, Nrf2 is inactive and mainly locates in the cytoplasm. In oxidative stress status, Nrf2 may quickly translocate into nucleus to regulate the expression of downstream peroxiredoxin and increase the activity of antioxidation[20–22]**错误!超链接引用无效。错误!超链接引用无效。错误!超链接引用无效。**. The activation of Nrf2 could obviously promote HO-1 activity and partly inhibit oxidative stress. In the present study, the results suggested that naringin obviously activated Nrf2 signaling pathway and increased the expression and activity of its downstream target HO-1.

The article "Naringin Alleviates Diabetic Kidney Disease through Inhibiting Oxidative Stress and Inflammatory Reaction" was retracted in 2018. Reasons: false authorship; lack of ethics approval or compliance; ethical violations by an author.

So far a number of researches have also confirmed that DKD might be an inflammatory disease and inflammation promoted the progression of DKD[23, 24]**错误!超链接引用无效。错误!超链接引用无效。**. In the development of DKD, inflammatory cell infiltration is obvious in kidney tissue with increased levels of pro-inflammatory cytokines in peripheral blood[25–27]**错误!超链接引用无效。错误!超链接引用无效。错误!超链接引用无效。**. It is effective to delay the development of DKD by controlling inflammatory response[28, 29]**错误!超链接引用无效。错误!超链接引用无效。**. Recent studies have found that the increased production of ROS induced by high glucose was the main cause of inflammatory reaction and inflammation would which, in turn, prompt oxidative stress[30, 31]**错误!超链接引用无效。错误!超链接引用无效。**. Oxidative stress and inflammatory reaction are of mutual cause-effect and mutual promotion relationship in the progression of DKD. Our results also confirmed the protective effect of naringin against inflammatory reaction in diabetic rats in vivo and high glucose-induced HBZY-1 cells in vitro.

Nuclear factor-kappa B(NF-κ B) is a transcription factor broadly expressed in tissues, which is the key molecule in inflammation reaction in DKD[32]. NF-κ B could be activated by various signaling pathways. The phosphorylation and degradation of I κ B α plays pivotal role in NF-κ B activation[33]. The activation of NF-κ B is obviously increased in kidney of diabetic animals, which promotes the hyperplasia of mesangial cells[34]. In the oxidative stress status, ROS could promote the pro-inflammatory cytokines production and aggravate the inflammatory response by activating NF-κ B[35, 36]**错误!超链接引用无效。错误!超链接引用无效。**. The inhibition of NF-κ B signaling pathway could significantly alleviate oxidative stress injury and inflammatory reaction induced by high glucose[37]. The activation of Nrf2 could enhance the antioxidant enzymes expression via inhibiting NF-κ B activation, which plays important roles in restraining oxidative stress injury and inflammatory reaction in DKD[38]. In this study, we demonstrated that naringin inhibited the activation of NF-κ B signaling pathway induced by STZ or high glucose, suggesting that NF-κ B was involved in the protective effect of naringin against DKD.

In order to better investigate the protective effect of naringin, the role of naringenin, aglycone of naringin, was also observed in vitro. Study by Zuo et al showed that naringin and total naringenin were rapidly and widely distributed to all the tissues except brain in rats after oral administration of naringin[39]. An earlier research has demonstrated that plasma concentration-time profiles of naringin were found to increase quickly and decline rapidly within 2 h in rats and naringenin and naringenin glucuronide were identified as two metabolites of naringin in rats plasma[40]. So naringenin has close relation with naringin and the research on naringenin is considered to be significant. In our present study, the naringenin could inhibit high glucose-induced proliferation, inflammatory reactions and oxidative stress injury in vitro, which was consistent with the results of naringin.

The article "Naringin Alleviates Diabetic Kidney Disease through Inhibiting Oxidative Stress and Inflammatory Reaction" was retracted in 2018. Reasons: false authorship; lack of ethics approval or compliance; ethical violations by an author.

In conclusion, our study demonstrated that naringin improved renal function, decreased collagen formation and ECM accumulation, restrained oxidative stress injury and inflammatory reaction by inhibiting NF-κ B signaling pathway. Among several doses of naringin for in vivo study, our results demonstrated that 80 mg/kg is the dosage that worked best. Although the effects of naringin on DKD and the relative molecular mechanisms require further investigation, we could draw a conclusion that naringin has the potential to be used for treatment of DKD.

## Supporting Information

S1 Fig Naringenin suppressed high glucose-induced proliferation, inflammatory reaction and oxidative stress injury in HBZY-1 cells. (A) The molecular formula of naringenin is C15H12O5 and the molecular weight is 272.25. (B) The effect of naringenin on high glucose-induced proliferation in HBZY-1 cells was determined by MTT assay. Data were expressed as means±SD, n = 5. (C-F) The TNF-α, MCP-1, ICAM-1 and VCAM-1 levels in HBZY-1 cells were determined by ELISA assay. Data were expressed as means±SD, n = 3. (G) The ROS production in HBZY-1 cells was evaluated by flow cytometry and ROS generation rates were shown. Data were expressed as means±SD, n = 3. (F) The protein levels of NF-κ B, HO-1 and Nrf2 in HBZY-1 cells were determined by western blot.^a-d^ Means with different superscripts are significantly different (P< 0.05).
(TIF)

## References

[1] CrandallJP, KnowlerWC, KahnSE, MarreroD, FlorezJC, BrayGA, et al The prevention of type 2 diabetes. Nat Clin Pract Endocrinol Metab. 2008;4(7):382–93. Epub 2008/05/22. doi: 10.1038/ncpendmet0843 ncpendmet0843[pii]. ; PubMed Central PMCID: PMC2573045.1849322710.1038/ncpendmet0843PMC2573045

[2] BrownleeM. Biochemistry and molecular cell biology of diabetic complications. Nature. 2001;414(6865):813–20. Epub 2001/12/14. doi: 10.1038/414813a 414813a[pii]. .1174241410.1038/414813a

[3] BrennerBM, CooperME, de ZeeuwD, KeaneWF, MitchWE, ParvingHH, et al Effects of losartan on renal and cardiovascular outcomes in patients with type 2 diabetes and nephropathy. N Engl J Med. 2001;345(12):861–9. Epub 2001/09/22. doi: 10.1056/NEJMoa011161 .1156551810.1056/NEJMoa011161

The article "Naringin Alleviates Diabetic Kidney Disease through Inhibiting Oxidative Stress and Inflammatory Reaction" was retracted in 2018. Reasons: false authorship; lack of ethics approval or compliance; ethical violations by an author.

[4] KanwarYS, WadaJ, SunL, XieP, WallnerEI, ChenS, et al Diabetic nephropathy: mechanisms of renal disease progression. Exp Biol Med (Maywood). 2008;233(1):4–11. Epub 2007/12/25. 233/1/4 [pii] doi: 10.3181/0705-MR-134 .1815630010.3181/0705-MR-134

[5] BhartiS, RaniN, KrishnamurthyB, AryaDS. Preclinical evidence for the pharmacological actions of naringin: a review. Planta Med. 2014;80(6):437–51. Epub 2014/04/09. doi: 10.1055/s-0034-1368351 .2471090310.1055/s-0034-1368351

[6] JungUJ, LeemE, KimSR. Naringin: a protector of the nigrostriatal dopaminergic projection. Exp Neurobiol. 2014;23(2):124–9. Epub 2014/06/26. doi: 10.5607/en.2014.23.2.124 ; PubMed Central PMCID: PMC4065825.2496327610.5607/en.2014.23.2.124PMC4065825

[7] XuluS, Oroma OwiraPM. Naringin ameliorates atherogenic dyslipidemia but not hyperglycemia in rats with type 1 diabetes. J Cardiovasc Pharmacol. 2012;59(2):133–41. Epub 2011/10/04. doi: 10.1097/FJC.0b013e31823827a4 .2196415810.1097/FJC.0b013e31823827a4

[8] MahmoudAM, AshourMB, Abdel-MoneimA, AhmedOM. Hesperidin and naringin attenuate hyperglycemia-mediated oxidative stress and proinflammatory cytokine production in high fat fed/streptozotocin-induced type 2 diabetic rats. J Diabetes Complications. 2012;26(6):483–90. Epub 2012/07/20. doi: 10.1016/j.jdiacomp.2012.06.001 S1056-8727(12)00177-8 [pii]. .2280989810.1016/j.jdiacomp.2012.06.001

[9] ShinEJ, HurHJ, SungMJ, ParkJH, YangHJ, KimMS, et al Ethanol extract of the Prunus mume fruits stimulates glucose uptake by regulating PPAR-gamma in C2C12 myotubes and ameliorates glucose intolerance and fat accumulation in mice fed a high-fat diet. Food Chem. 2013;141(4):4115–21. Epub 2013/09/03. doi: 10.1016/j.foodchem.2013.06.059 S0308-8146(13)00836-4 [pii]. .2399359310.1016/j.foodchem.2013.06.059

[10] ChenJ, GuoR, YanH, TianL, YouQ, LiS, et al Naringin inhibits ROS-activated MAPK pathway in high glucose-induced injuries in H9c2 cardiac cells. Basic Clin Pharmacol Toxicol. 2014;114(4):293–304. Epub 2013/10/15. doi: 10.1111/bcpt.12153 .2411882010.1111/bcpt.12153

[11] KandhareAD, GhoshP, BodhankarSL. Naringin, a flavanone glycoside, promotes angiogenesis and inhibits endothelial apoptosis through modulation of inflammatory and growth factor expression in diabetic foot ulcer in rats. Chem Biol Interact. 2014;219:101–12. Epub 2014/06/01. doi: 10.1016/j.cbi.2014.05.012 S0009-2797(14)00170-7 [pii]. .2488002610.1016/j.cbi.2014.05.012

[12] MullenW, EdwardsCA, CrozierA. Absorption, excretion and metabolite profiling of methyl-, glucuronyl-, glucosyl- and sulpho-conjugates of quercetin in human plasma and urine after ingestion of onions. Br J Nutr. 2006;96(1):107–16. Epub 2006/07/28. S000711450600184X [pii]. .1686999810.1079/bjn20061809

The article "Naringin Alleviates Diabetic Kidney Disease through Inhibiting Oxidative Stress and Inflammatory Reaction" was retracted in 2018. Reasons: false authorship; lack of ethics approval or compliance; ethical violations by an author.

[13] FabreJ, BalantLP, DayerPG, FoxHM, VernetAT. The kidney in maturity onset diabetes mellitus: a clinical study of 510 patients. Kidney Int. 1982;21(5):730–8. Epub 1982/05/01. .710945910.1038/ki.1982.90

[14] SinghDK, WinocourP, FarringtonK. Oxidative stress in early diabetic nephropathy: fueling the fire. Nat Rev Endocrinol. 2011;7(3):176–84. Epub 2010/12/15. doi: 10.1038/nrendo.2010.212 nrendo.2010.212 [pii]. .2115120010.1038/nrendo.2010.212

[15] KashiharaN, HarunaY, KondetiVK, KanwarYS. Oxidative stress in diabetic nephropathy. Curr Med Chem. 2010;17(34):4256–69. Epub 2010/10/14. BSP/CMC/E-Pub/ 265 [pii]. ; PubMed Central PMCID: PMC3708695.2093981410.2174/092986710793348581PMC3708695

[16] KitadaM, KumeS, ImaizumiN, KoyaD. Resveratrol improves oxidative stress and protects against diabetic nephropathy through normalization of Mn-SOD dysfunction in AMPK/SIRT1-independent pathway. Diabetes. 2011;60(2):634–43. Epub 2011/01/29. doi: 10.2337/db10-0386 60/2/634 [pii]. ; PubMed Central PMCID: PMC3028365.2127027310.2337/db10-0386PMC3028365

[17] MatoughFA, BudinSB, HamidZA, AlwahaibiN, MohamedJ. The role of oxidative stress and antioxidants in diabetic complications. Sultan Qaboos Univ Med J. 2012;12(1):5–18. Epub 2012/03/01. ; PubMed Central PMCID: PMC3286717.2237525310.12816/0003082PMC3286717

[18] Kedziora-KornatowskaK, SzramS, KornatowskiT, Szadujkis-SzadurskiL, KedzioraJ, BartoszG. Effect of vitamin E and vitamin C supplementation on antioxidative state and renal glomerular basement membrane thickness in diabetic kidney. Nephron Exp Nephrol. 2003;95(4):e134–43. Epub 2003/12/25. 74840 74840 [pii]. .1469426710.1159/000074840

[19] BhattiF, MankheyRW, AsicoL, QuinnMT, WelchWJ, MaricC. Mechanisms of antioxidant and pro-oxidant effects of alpha-lipoic acid in the diabetic and nondiabetic kidney. Kidney Int. 2005;67(4):1371–80. Epub 2005/03/23. KID214 [pii] doi: 10.1111/j.1523-1755.2005.00214.x .1578008910.1111/j.1523-1755.2005.00214.x

[20] BuckleyBJ, LiS, WhortonAR. Keap1 modification and nuclear accumulation in response to S-nitrosocysteine. Free Radic Biol Med. 2008;44(4):692–8. Epub 2007/12/08. S0891-5849(07)00754-X [pii] doi: 10.1016/j.freeradbiomed.2007.10.055 ; PubMed Central PMCID: PMC2267934.1806293110.1016/j.freeradbiomed.2007.10.055PMC2267934

[21] KangMI, KobayashiA, WakabayashiN, KimSG, YamamotoM. Scaffolding of Keap1 to the actin cytoskeleton controls the function of Nrf2 as key regulator of cytoprotective phase 2 genes. Proc Natl Acad Sci U S A. 2004;101(7):2046–51. Epub 2004/02/07. doi: 10.1073/pnas.0308347100 0308347100 [pii]. ; PubMed Central PMCID: PMC357049.1476489810.1073/pnas.0308347100PMC357049

The article "Naringin Alleviates Diabetic Kidney Disease through Inhibiting Oxidative Stress and Inflammatory Reaction" was retracted in 2018. Reasons: false authorship; lack of ethics approval or compliance; ethical violations by an author.

[22] ShenG, JeongWS, HuR, KongAN. Regulation of Nrf2, NF-kappaB, and AP-1 signaling pathways by chemopreventive agents. Antioxid Redox Signal. 2005;7(11–12):1648–63. Epub 2005/12/17. doi: 10.1089/ars.2005.7.1648 .1635612710.1089/ars.2005.7.1648

[23] Luis-RodriguezD, Martinez-CastelaoA, GorrizJL, De-AlvaroF, Navarro-GonzalezJF. Pathophysiological role and therapeutic implications of inflammation in diabetic nephropathy. World J Diabetes. 2012;3(1):7–18. Epub 2012/01/19. doi: 10.4239/wjd.v3.i1.7 ; PubMed Central PMCID: PMC3258536.2225394110.4239/wjd.v3.i1.7PMC3258536

[24] RiveroA, MoraC, MurosM, GarciaJ, HerreraH, Navarro-GonzalezJF. Pathogenic perspectives for the role of inflammation in diabetic nephropathy. Clin Sci (Lond). 2009;116(6):479–92. Epub 2009/02/10. doi: 10.1042/CS20080394 CS20080394 [pii]. .1920005710.1042/CS20080394

[25] TeschGH. Macrophages and diabetic nephropathy. Semin Nephrol. 2010;30(3):290–301. Epub 2010/07/14. doi: 10.1016/j.semnephrol.2010.03.007 S0270-9295(10)00057-4 [pii]. .2062067310.1016/j.semnephrol.2010.03.007

[26] KingGL. The role of inflammatory cytokines in diabetes and its complications. J Periodontol. 2008;79(8 Suppl):1527–34. Epub 2008/09/04. doi: 10.1902/jop.2008.080246 .1867300710.1902/jop.2008.080246

[27] TaslipinarA, YamanH, YilmazMI, DemirbasS, SaglamM, TaslipinarMY, et al The relationship between inflammation, endothelial dysfunction and proteinuria in patients with diabetic nephropathy. Scand J Clin Lab Invest. 2011;71(7):606–12. Epub 2011/08/26. doi: 10.3109/00365513.2011.598944 .2186405410.3109/00365513.2011.598944

[28] Sanchez-NinoMD, BozicM, Cordoba-LanusE, ValchevaP, GraciaO, IbarzM, et al Beyond proteinuria: VDR activation reduces renal inflammation in experimental diabetic nephropathy. Am J Physiol Renal Physiol. 2012;302(6):F647–57. Epub 2011/12/16. doi: 10.1152/ajprenal.00090.2011 ajprenal.00090.2011 [pii]. .2216900910.1152/ajprenal.00090.2011

[29] WuJ, GuanTJ, ZhengS, GrosjeanF, LiuW, XiongH, et al Inhibition of inflammation by pentosan polysulfate impedes the development and progression of severe diabetic nephropathy in aging C57B6 mice. Lab Invest. 2011;91(10):1459–71. Epub 2011/08/03. doi: 10.1038/labinvest.2011.93 labinvest201193 [pii]. .2180823810.1038/labinvest.2011.93

[30] ElmarakbyAA, SullivanJC. Relationship between oxidative stress and inflammatory cytokines in diabetic nephropathy. Cardiovasc Ther. 2012;30(1):49–59. Epub 2010/08/20. doi: 10.1111/j.1755-5922.2010.00218.x CDR218 [pii]. .2071875910.1111/j.1755-5922.2010.00218.x

[31] Lopes de FariaJB, SilvaKC, Lopes de FariaJM. The contribution of hypertension to diabetic nephropathy and retinopathy: the role of inflammation and oxidative stress. Hypertens Res. 2011;34(4):413–22. Epub 2011/01/14. doi: 10.1038/hr.2010.263 hr2010263 [pii]. .2122878310.1038/hr.2010.263

The article "Naringin Alleviates Diabetic Kidney Disease through Inhibiting Oxidative Stress and Inflammatory Reaction" was retracted in 2018. Reasons: false authorship; lack of ethics approval or compliance; ethical violations by an author.

[32] YiB, HuX, ZhangH, HuangJ, LiuJ, HuJ, et al Nuclear NF-kappaB p65 in peripheral blood mononuclear cells correlates with urinary MCP-1, RANTES and the severity of type 2 diabetic nephropathy. PLoS One. 2014;9(6):e99633 Epub 2014/06/18. doi: 10.1371/journal.pone.0099633 PONE-D-13-37392 [pii]. ; PubMed Central PMCID: PMC4061032.2493686610.1371/journal.pone.0099633PMC4061032

[33] HanJG, GuptaSC, PrasadS, AggarwalBB. Piperlongumine chemosensitizes tumor cells through interaction with cysteine 179 of IkappaBalpha kinase, leading to suppression of NF-kappaB-regulated gene products. Mol Cancer Ther. 2014;13(10):2422–35. Epub 2014/08/02. doi: 10.1158/1535-7163.MCT-14-0171 1535-7163.MCT-14-0171 [pii]. .2508296110.1158/1535-7163.MCT-14-0171

[34] GuijarroC, EgidoJ. Transcription factor-kappa B (NF-kappa B) and renal disease. Kidney Int. 2001;59(2):415–24. Epub 2001/02/13. kid516 [pii] doi: 10.1046/j.1523-1755.2001.059002415.x .1116892310.1046/j.1523-1755.2001.059002415.x

[35] CalcuttNA, CooperME, KernTS, SchmidtAM. Therapies for hyperglycaemia-induced diabetic complications: from animal models to clinical trials. Nat Rev Drug Discov. 2009;8(5):417–29. Epub 2009/05/01. doi: 10.1038/nrd2476 nrd2476[pii]. .1940431310.1038/nrd2476PMC7097138

[36] KernTS. Contributions of inflammatory processes to the development of the early stages of diabetic retinopathy. Exp Diabetes Res. 2007;2007:95103 Epub 2008/02/16. doi: 10.1155/2007/95103 ; PubMed Central PMCID: PMC2216058.1827460610.1155/2007/95103PMC2216058

[37] KumarA, NegiG, SharmaSS. Suppression of NF-kappaB and NF-kappaB regulated oxidative stress and neuroinflammation by BAY 11–7082 (IkappaB phosphorylation inhibitor) in experimental diabetic neuropathy. Biochimie. 2012;94(5):1158–65. Epub 2012/02/22. doi: 10.1016/j.biochi.2012.01.023 S0300-9084(12)00041-7 [pii]. .2234222410.1016/j.biochi.2012.01.023

[38] LyuJH, LeeGS, KimKH, KimHW, ChoSI, JeongSI, et al ent-kaur-16-en-19-oic Acid, isolated from the roots of Aralia continentalis, induces activation of Nrf2. J Ethnopharmacol. 2011;137(3):1442–9. Epub 2011/09/03. doi: 10.1016/j.jep.2011.08.024 S0378-8741(11)00597-6 [pii]. ; PubMed Central PMCID: PMC3616193.2188477810.1016/j.jep.2011.08.024PMC3616193

[39] ZouW, YangC, LiuM, SuW. Tissue distribution study of naringin in rats by liquid chromatography-tandem mass spectrometry. Arzneimittelforschung. 2012;62(4):181–6. Epub 2012/01/25. doi: 10.1055/s-0031-1299746 .2227084410.1055/s-0031-1299746

The article "Naringin Alleviates Diabetic Kidney Disease through Inhibiting Oxidative Stress and Inflammatory Reaction" was retracted in 2018. Reasons: false authorship; lack of ethics approval or compliance; ethical violations by an author.

[40] FangT, WangY, MaY, SuW, BaiY, ZhaoP. A rapid LC/MS/MS quantitation assay for naringin and its two metabolites in rats plasma. J Pharm Biomed Anal. 2006;40(2):454–9. Epub 2006/01/13. S0731-7085(05)00497-8 [pii] doi: 10.1016/j.jpba.2005.07.031 .1640644210.1016/j.jpba.2005.07.031

